# Identifying Obstructive Sleep Apnea Syndrome-Associated Genes and Pathways through Weighted Gene Coexpression Network Analysis

**DOI:** 10.1155/2022/3993509

**Published:** 2022-01-29

**Authors:** Yan Li, Li Li, Hua Zhao, Xiwen Gao, Shanqun Li

**Affiliations:** ^1^Department of Respiratory, Minhang Hospital, Fudan University, 170 Xinsong Road, Minhang District, Shanghai, China 201199; ^2^Department of Pulmonary Medicine, Minhang Branch, Zhongshan Hospital, Fudan University, 180 Fenglin Rd, Shanghai, China 200032

## Abstract

**Background:**

Obstructive sleep apnea syndrome (OSAS) is the most common type of sleep apnea disorder. The disease seriously affects the patient's respiratory system. At present, the prognosis of the disease is poor and there is a lack of effective treatments. Therefore, it is urgent to explore its pathogenesis and treatment methods.

**Method:**

We downloaded a set of expression profile data from GSE75097 related to OSAS based on the Gene Expression Omnibus (GEO) database and selected the representative differentially expressed genes (DEGs) from the sample of the GSE75097 dataset. WGCNA was used to find genes related to OSAS and obtain coexpression modules. The Gene Ontology (GO) function and the Kyoto Encyclopedia of Genes and Genomes (KEGG) pathway were used to analyze genes from key modules. Finally, Cytoscape software was used to construct a protein-protein interaction (PPI) network and analyze the hub genes.

**Result:**

We obtained a total of 7565 DEGs. Through WGCNA, we got four coexpression modules and the modules most related to OSAS were green-yellow, magenta, purple, and turquoise, and we screened out eight hub genes (DDX46, RNF115, COPA, FBXO4, PA2G4, NHP2L1, CDC20, and PCNA). GO and KEGG analyses indicated that the key modules were mainly enriched in tRNA modification, nucleobase metabolic process, DNA ligation, regulation of cellular component movement, basal transcription factors, Huntington disease, and vitamin digestion and absorption.

**Conclusion:**

These pathways and hub genes can facilitate understanding the molecular mechanism of OSAS and provide a meaningful reference for finding biological targets of OSAS treatment.

## 1. Background

Obstructive sleep apnea syndrome (OSAS) is a sleep breathing disorder with unknown etiology, which is manifested as upper airway obstruction, apnea during sleep, hypoxia, snoring, and daytime sleepiness [1, 2]. The disease often occurs in the obese and the elderly, and it is also common in children with sleep-disordered breathing [3]. It is worth noting that OSAS can also affect the patient's cardiovascular system, respiratory system, cerebrovascular, central nervous system, endocrine, sexual function, kidney, blood system, and digestive system and even threaten life [4]. Currently, adenoid and tonsillectomy are the main treatments for most children with OSAS [5]. In addition, the Continuous Positive Airway Pressure (CPAP) is also a device specially developed and manufactured for newborns used for respiratory support [6].

Genomics is aimed at systematically characterizing and quantifying all genes in an organism and studying the relationship among them and their impact on the organism [7]. Genome technology usually includes high-throughput sequencing technology, genome editing technology, and metagenomic technology [8]. Goldfield et al. believe that genomic technology can help to better understand disease subtypes and characteristics at the human level and provide individual-level diagnosis and personalized treatment [9]. Through comprehensive bioinformatics analysis, Gui et al. identified the candidate markers related to the pathology of Alzheimer's disease (AD) and provided comprehensive insight into understanding AD's pathogenesis and potential new therapeutic targets [10]. With the further development of genome technology, the integration and reanalysis of data kept in public databases can give vital insights for a new study, as well as vast prospects for illness target research [11].

This time, we conducted a series of bioinformatics analyses on 48 samples in the GSE75097 dataset based on weighted gene coexpression network analysis (WGCNA) [12]. Firstly, differentially expressed genes (DEGs) were screened out from the samples, and on this basis, key modules highly related to OSAS were determined through WGCNA [13]. After that, Gene Ontology (GO) function and Kyoto Encyclopedia of Genes and Genomes (KEGG) pathway enrichment analyses were performed on DEGs in key modules [14], and protein-protein interaction (PPI) network construction and hub gene screening were performed again on modules with a large number of genes [15]. The above methods will help us find OSAS-related therapeutic targets.

## 2. Material and Methods

### 2.1. Acquisition of Microarray Dataset

The microarray dataset GSE75097 provided was downloaded from the Gene Expression Omnibus (GEO, https://www.ncbi.nlm.nih.gov/geo/) database. We analyzed whole-genome gene expression profiles of 48 patients with sleep-disordered breathing stratified into four groups: 6 primary snoring (PS) samples, 16 moderate to severe OSA (MSO) samples, 12 very severe OSA (VSO) samples, and 14 very severe OSA patients with long-term CPAP treatment (VSOC) samples. After that, we used Robust Multiarray Average (RMA) algorithm to process the above 48 samples and filtered the subsequent WGCNA data through nsFilter algorithm.

### 2.2. Construction of WGCNA and Identification of Key Modules

WGCNA is a freely accessible R package that identifies the gene set of interest based on the information of thousands of the most changing genes or all genes and performs significant association analysis with phenotypes to construct a gene coexpression network. In this study, we determined the best soft threshold based on this method to make the gene network follow the scale-free distribution. Then, we defined the gene coexpression correlation matrix, constructed a hierarchical clustering tree of gene modules according to the formed adjacency function, and finally determined the modules most relevant to OSAS based on the heat map for subsequent bioinformatics analysis.

### 2.3. Function Enrichment Analysis of Key Modules

The Database for Annotation, Visualization, and Integrated Discovery (DAVID, https://david.ncifcrf.gov/) is an online analysis tool released in 2003. Like other similar analysis tools, it associates the genes in the input list with the biological annotation term and then uses statistical methods to find the most significantly enriched biological annotations. GO is a database that defines and describes the functions of genes and proteins. It is divided into three categories: molecular function (MF), biological process (BP), and cellular component (CC). The KEGG database has 17 subdatabases in 4 categories, including genome, chemistry, and system function information, and KEGG pathway is usually used to store information about gene pathways in different species. This time, we performed enrichment analysis on the genes in the key modules based on the DAVID database.

### 2.4. Acquisition of DEGs of Key Modules and Construction of PPI Networks

After performing functional enrichment analysis on the genes obtained in the key modules, the DEGs in the modules were screened by GEO2R (https://www.ncbi.nlm.nih.gov/geo/geo2r/). Later, in order to find genes related to OSAS, we used the Search Tool for the Retrieval of Interacting Genes (STRING, https://string-db.org/) database and Cytoscape (https://www.cytoscape.org/) software to design the PPI network of the two modules with the largest number of DEGs. Finally, according to the Molecular Complex Detection (MCODE) method, the genes with the highest degree value were identified as the hub genes in this study.

## 3. Results

### 3.1. Data Processing

We downloaded the GSE75097 microarray dataset from the GEO database, which involved a total of 48 samples. The original files were background corrected, normalized, and summarized by the RMA algorithm of the R language, and a total of 7565 DEGs were obtained for subsequent WGCNA analysis (Figure 1).

### 3.2. Construction of WGCNA Related to OSAS Modules

After obtaining 7565 DEGs from 48 samples, WGCNA was constructed on this basis. First, we determined the optimal soft threshold (*β* = 6) that conformed to the scale-free topology network to define the adjacency matrix (Figure 2(a)). After that, we clustered the genes with the same expression into the same module to construct a modular gene tree diagram (Figure 2(b)). Then, we got 13 different gene modules, which were divided into two clusters, all related to OSAS (Figure 3(a)). Finally, we selected 9 modules to construct the eigengene adjacency heat map (Figure 3(b)). It should be noted that the gray module contained all genes that were not involved in clustering and would not be analyzed.

### 3.3. GO Enrichment Analysis of the Genes in Key Modules

According to Figures 4(a)–4(d), in GO, the genes of the green-yellow module were enriched in intra-Golgi vesicle-mediated transport, tRNA modification, RNA modification, negative regulation of transcription regulatory region DNA binding, positive regulation of smoothened signaling pathway and extrinsic apoptotic signaling pathway via death domain receptors, etc. The genes in the magenta module were enriched in the nucleobase metabolic process, pyrimidine nucleobase metabolic process, tRNA modification, negative regulation of JNK cascade and stress-activated MAPK cascade, low-density lipoprotein particle receptor catabolic process, chylomicron assembly, very-low-density lipoprotein particle assembly, etc. The genes in the purple module were enriched in DNA ligation, pteridine-containing compound biosynthetic process, inositol lipid-mediated signaling, positive regulation of protein complex disassembly, phosphatidylinositol phosphorylation, regulation of telomerase RNA localization to Cajal body, acyl-CoA biosynthetic process, etc. In addition, genes in turquoise modules were also enriched in regulation of cellular component movement, mitochondrial ATP synthesis-coupled proton transport, protein localization to Golgi apparatus, regulation of microtubule-based process, cristae formation, ATP synthesis-coupled proton transport, purine ribonucleoside triphosphate biosynthetic process, etc.

### 3.4. KEGG Enrichment Analysis of the Genes in Key Modules

According to the results of the enrichment of KEGG, it was not difficult to find that the genes in the green-yellow module were enriched in vasopressin-regulated water reabsorption, basal transcription factors, propanoate metabolism, selenocompound metabolism, thyroid cancer, other types of O-glycan biosynthesis, and other pathways (Figure 5(a)). The genes in the magenta module were enriched in Huntington's disease, pyrimidine metabolism, cardiac muscle contraction, oxidative phosphorylation, Parkinson's disease, fat digestion and absorption, nonalcoholic fatty liver disease (NAFLD), and other pathways (Figure 5(b)). The genes in the purple module were enriched in vitamin digestion and absorption, folate biosynthesis, fatty acid biosynthesis, RNA polymerase, fatty acid degradation, base excision repair, etc. (Figure 5(c)). Genes in the turquoise module were enriched in alpha-linolenic acid metabolism, glycosylphosphatidylinositol- (GPI-) anchor biosynthesis, maturity onset diabetes of the young, collecting duct acid secretion, linoleic acid metabolism, citrate cycle (TCA cycle), etc. (Figure 5(d)).

### 3.5. DEGs and Hub Genes of Key Modules

Figure 6 shows the heat map of DEGs in the four key modules. Among them, the number of DEGs in the green-yellow module was 846, the number of DEGs in the magenta module was 206, that in the purple module was 2743, and that in the turquoise module was 152. Next, we selected the two modules with the largest number of DEGs to construct the PPI network. It could be seen from Figure 7(a) that the PPI network of the yellow-green module consisted of 30 nodes and 101 edges; DDX46, RNF115, COPA, and FBXO4 had the same degree value, all being 8. In addition, we also constructed three different PPI networks based on the DEGs in the purple module. The degree values of the hub genes (PA2G4, NHP2L1) in the PPI network (39 nodes and 681 edges) in Figure 7(b) were all 94, and the hub gene in the PPI network (56 nodes and 523 edges) in Figure 7(c) was CDC20 (degree = 33). The hub gene obtained in the PPI network (49 nodes and 398 edges) in Figure 7(d) was PCNA (degree = 23). The detailed information regarding the hub genes is shown in Table 1.

## 4. Discussion

Herein, we conduct a series of bioinformatics analyses on 48 samples in the GSE75097 dataset based on WGCNA. In the functional enrichment analysis of GO, the genes of these modules are mainly enriched in biological processes related to epigenetics, including RNA modification, DNA binding and tRNA, nucleobase metabolic process, pyrimidine nucleobase metabolic process, negative regulation of JNK cascade, and tRNA modification. The so-called epigenetics refers to heritable phenotypic changes without those in DNA sequence [16]. In recent years, hypoxia-mediated epigenetic regulation has had a major function in the mechanism of OSAS [17]. Under chronic intermittent hypoxia-reoxygenation circumstances, the epigenetic process influences the adaptive potential and phenotypic variability, which contributes to the development of numerous deleterious effects of OSAS [18, 19].

In addition, chemical modification of nucleobases functions importantly in different levels of gene expression control. It includes modulating tRNA bases to regulate translation or cytosine methylation and demethylation in the promoter region to silence and reactivate genes. Chen et al. speculated that hypomethylation of the six gene promoter regions implicated in the NPR2 and SP140 pathways may play a crucial role in the establishment of the OSAS phenotype of excessive daytime sleepiness [20]. Nevertheless, chronic IHR may trigger these DNA methylation changes, leading to frequent hypoxia and lethargy phenotypes in OSAS [21].

In the KEGG pathway analysis, the enrichment results in the green-yellow module are not highly correlated with OSAS. In the magenta module and the purple module, reports are showing the roles of cardiac muscle contraction, nonalcoholic fatty liver disease (NAFLD), and folate in breathing. Apnea during dynamic exercise activates the human muscle metabolism reflex [22]. During apnea, the decrease in O_2_ delivery to the working muscles triggers the muscle metabolic reflex. The activation of the muscle metabolic reflex is one of the potential mechanisms of the blood pressure response induced by significant apnea [23]. The study by Kuo et al. showed that maximum expiratory apnea increased the kinetic energy of the heart which was calculated from shock cardiography BCG and seismocardiography SCG, as well as sympathetic nerve activity [24]. Therefore, cardiac contraction is closely related to apnea.

Cyanide is a toxin that may be found in a variety of foods, as well as home and industrial items, some ready-made products included [25]. The combination of cyanide and cytochrome oxidase can paralyze cell respiration [26]. The signs and symptoms of cyanide poisoning may include abnormal breathing, that is, shortness of breath and dyspnea that progress to respiratory depression and apnea [27]. Therefore, oxidative phosphorylation is an inducing factor of apnea, and attention should be paid to its combination with cyanide [28]. OSAS mostly occurs in patients with Parkinson's disease (PD) and nonalcoholic fatty liver disease (NAFLD). However, the relationship between OSAS and PD and NAFLD still needs further research to prove its pathogenic molecular mechanism. Relevant studies have indicated folic acid deficiency is substantially associated with obstructive sleep apnea in women [29].

The hub genes we selected from green-yellow module and purple module are reported to correlate with breath and disease related to the lung. There are reports on the relationship between RNF115 and lung adenocarcinoma (LAC). RNF115-mediated p53 ubiquitination can act as the marker of the prognosis of patients with LAC [30]. RNF115 induces a significant arrest of the G1 phase of LAC cells to achieve the function of inhibiting cell viability *in vitro*, further reducing tumor proliferation in xenograft models. These findings suggest that RNF115 might be a novel predictive biomarker and that the RNF115-p53 axis could be a target for LAC therapy. The cuffed oropharyngeal airway (COPA) is a modified Guedel-type oral airway with a cuff on the end. Propofol and sevoflurane are equally effective in promoting the placement of COPA [31]. However, propofol usually causes apnea, which is complicated by the poor sealing effect of COPA on the airway. At the same time, sevoflurane allows spontaneous breathing to continue and provides sufficient pharynx seal immediately after that COPA is placed, so it may be advantageous when apnea is not required. Propofol and sevoflurane can promote the placement of COPA to treat obstructive sleep-disordered breathing. Studies have confirmed that several tumor aggressiveness markers like PCNA have high expression, providing molecular evidence for the relationship between apnea and cancer. PCNA is a biomarker that identifies the relationship between apnea and cancer [32]. The results of this study need further experimental verification. In future research, we will explore the specific mechanism of the hub gene in the pathogenesis of OSAS. The correlation between the expression level of the hub gene and the clinical parameters of OSAS patients needs to be further explored.

In conclusion, our analysis results show that the genes in the selected key modules are mainly enriched in epigenetics, DNA methylation, and nucleobases. The hub genes (RNF115, COPA, and PCNA) selected from the key modules are biomarkers related to OSAS, which provides useful information for the therapies of diseases related to OSAS. However, five of these hub genes have not been studied in OSAS, but they are all important hub genes for understanding OSAS, predicting prognosis, and developing precise therapies.

## Figures and Tables

**Figure 1:** Heat map of the GSE75097 dataset. One column is a sample, and one row is a gene.

**Figure 2:** WGCNA construction. (a) The left picture is used to determine the optimal soft threshold, and the right picture shows the network connectivity under different soft thresholds. (b) Gene dendrogram and module colors.

**Figure 3:** Modules in WGCNA. (a) Cluster map of 13 eigengene modules. (b) Eigengene adjacency heat map of 9 modules.

**Figure 4:** GO function enrichment results. (a) Green-yellow module. (b) Magenta module. (c) Purple module. (d) Turquoise module.

**Figure 5:** KEGG pathway enrichment results. (a) Green-yellow modules. (b) Magenta module. (c) Purple module. (d) Turquoise modules.

**Figure 6:** Heat map of four modules. (a) Green-yellow module with 846 DEGs. (b) Magenta module with 206 DEGs. (c) Purple module with 2743 DEGs. (d) Turquoise module with 152 DEGs.

**Figure 7:** PPI network of green-yellow and purple modules. (a) Green-yellow module, hub genes are DDX46, RNF115, COPA, and FBXO4. (b–d) Purple module, hub genes are PA2G4, NHP2L1, CDC20, and PCNA.

**Table 1:** The hub genes with higher degrees of PPI network of OSAS.

Gene symbol	Description	Degree	Module
DDX46	DEAD-box helicase 46	8	Green-yellow
RNF115	Ring finger protein 115	8	Green-yellow
COPA	Coatomer subunit *α*	8	Green-yellow
FBXO4	F-box protein 4	8	Green-yellow
PA2G4	Proliferation-associated 2G4	94	Purple
NHP2L1	U4/U6 small nuclear ribonucleoprotein	94	Purple
CDC20	Cell division cycle 20	33	Purple
PCNA	Proliferating cell nuclear antigen	23	Purple

## Data Availability

All data analyzed during this study are obtained from published article or are available from the corresponding author on reasonable request.
